This article has been retracted.

# Electroacupuncture attenuates cervical spinal cord injury following cerebral ischemia/reperfusion in stroke-prone renovascular hypertensive rats

**DOI:** 10.3892/etm.2014.1619

**Published:** 2014-03-12

**Authors:** FENG TAN, JIE CHEN, YANGUI LIANG, MINHUA GU, YANPING LI, XUEWEN WANG, DI MENG

**Affiliations:** 1 Department of Neurology, Foshan Hospital of Traditional Chinese Medicine, Guangzhou University of Chinese Medicine, Foshan, Guangdong 528000, P.R. China; 2 Department of Chinese Medicine, Dongsheng Hospital, Guangzhou, Guangdong 510120, P.R. China

**Keywords:** cerebral ischemia, cervical spinal cord, neuron, stroke-prone renovascular hypertensive rats

## Abstract

Cerebral ischemia induces injury, not only in the ischemic core and surrounding penumbra tissues, but also in remote areas such as the cervical spinal cord. The aim of the present study was to determine the effects of electroacupuncture (EA) on cervical spinal cord injury following cerebral ischemia/reperfusion in stroke-prone renovascular hypertensive (RHRSP) rats. The results demonstrated that neuronal loss, which was assayed by Nissl staining in the cervical spinal cords of RHRSP rats subjected to transient middle cerebral artery occlusion (MCAO), was markedly decreased by EA stimulation at the GV20 (Baihui) and GV14 (Dazhui) acupoints compared with that in rats undergoing sham stimulation. Quantitative polymerase chain reaction and western blot analysis demonstrated that EA stimulation blocked the MCAO-induced elevated protein expression levels of glial fibrillary acidic protein and amyloid precursor protein in the cervical spinal cord at days 24 and 48. To further investigate the mechanism underlying the neuroprotective role of EA stimulation, the protein expression levels of Nogo-A and Nogo-66 receptor-1 (NgR1), two key regulatory molecules for neurite growth, were recorded in each group. The results revealed that EA stimulation reduced the MCAO-induced elevation of Nogo-A and NgR1 protein levels at day 14 and 28 in RHRSP rats. Therefore, the results demonstrated that EA reduced cervical spinal cord injury following cerebral ischemia in RHRSP rats, indicating that EA has the potential to be developed as a therapeutic treatment agent for cervical spinal cord injury following stroke.

## Introduction

Cerebral ischemia induces neuronal cell death at the infarct core and secondary neuronal injury in the surrounding hypoperfused penumbra region, in addition to injuring the remote cervical spinal cord with which it is connected (1). Neuronal loss is topographically associated with axonal degeneration and is further induced by remote injury (2). The mechanisms underlying remote injury remain unclear and no treatment is yet available to reduce remote neuronal loss following cerebral ischemia.

Nogo-A is an inhibitor of neurite growth and is regulated by two inhibitory domains: 66-amino acid region (Nogo-66) and the N-terminal region (amino-Nogo). While amino-Nogo is important in axonal regeneration, sprouting and new network formation (3–5), Nogo-66 inhibits activity-dependent axonal growth by binding to the Nogo-66 receptor-1 (NgR1) (5). In turn, the NgR1 competitive antagonist, NEP1-40 (Nogo-66 residues 1–40), blocks this inhibitory effect (6). Notably, antibodies against Nogo-A improve neurological outcomes following ischemic stroke in adult rats (7). However, the role of Nogo-A and NgR1 in regulating remote alteration of the cervical spinal cord following cerebral ischemia remains unknown.

Traditionally, electroacupuncture (EA) therapy is recommended as a complementary method for pain relief and stroke rehabilitation (8). EA has been reported to improve neurological outcomes in animal models of cerebral ischemia/reperfusion (I/R) (9–11). Previously, we revealed that EA is able to protect neurons against I/R injury in stroke-prone renovascular hypertensive (RHRSP) rats and identified evidence that this process may be associated with the downregulation of Nogo-A (12,13). However, to date, there is little evidence available with regard to the efficacy of EA in the reduction of remote neuronal cell loss in the cervical spinal cord following cerebral ischemia.

In the present study, EA was used to stimulate the GV20 (Baihui) and GV14 (Dazhui) acupoints in order to investigate the neuroprotective role of EA in the cervical spinal cord following cerebral ischemia in RHRSP rats. In addition, changes in the expression of Nogo-A and NgR1 were evaluated to investigate the possible molecular mechanism.

## Materials and methods

### Ethics statement

All animal treatments were conducted in strict accordance with international ethical guidelines and the National Institutes of Health Guide for the Care and Use of Laboratory Animals (eighth edition, 2011). Experiments were performed with the approval of the Institutional Animal Care and Use Committee of Guangzhou University of Chinese Medicine (Foshan, China).

### Animals

Animals were provided by the Animal Center of the Guangzhou University of Chinese Medicine, in accordance with the Principles of Laboratory Animal Care, Guangzhou University of Chinese Medicine. In total, 300 male Sprague-Dawley rats (age, 30 days; weight, 70±20 g) were acclimated to laboratory conditions (temperature, 25±1°C; humidity, 65±5%; 12 h light/dark cycle; food and water, *ad libitum*) for three days prior to experimentation. Every effort was made to minimize the number of animals used and their suffering.

### Model of RHRSP

An RHRSP model was established, as previously described (14). Briefly, animals underwent renal artery constriction surgery using the two-kidney two-clip method. Under anesthesia [36 mg/kg sodium pentobarbital (3%) delivered intraperitoneally], a median longitudinal incision was made in the abdominal skin and the roots of the bilateral renal arteries were constricted by placing ring-shaped silver clips (inner diameter, 0.30 mm) to induce hypertension. Systolic blood pressure was measured in pre-warmed (37°C for 15 min), conscious rats using an indirect tail-cuff sphygmomanometer (MRB-IIIA; Shanghai Institute of Hypertension, Shanghai, China). Hypertension developed gradually in the majority of animals and became steady within eight weeks. Following surgery, the rats were transferred to an intensive care incubator in which the temperature was maintained at 37°C until the animals woke up completely. Subcutaneous injections of ketoprofen and twice daily monitoring of the rats’ well-being and surgical wound care were provided as postoperative care. For an immediate humane endpoint, the rats were administered chemical euthanasia (intraperitoneal injection of 200 mg/kg pentobarbital) prior to sacrifice.

### Transient middle cerebral artery occlusion (MCAO) model

Hypertensive rats (age, 12 weeks; weight, 350–500 g) without stroke symptoms and with a systolic blood pressure of >180 mmHg were used for the induction of cerebral ischemia. Rats were subjected to transient MCAO, as previously described (15). Briefly, a 4-cm length 4–0 surgical monofilament nylon suture coated with silicon was inserted from the external carotid artery into the internal carotid artery and further advanced to the Circle of Willis to occlude the origin of the right middle cerebral artery. After 2 h of ischemia, the intraluminal suture was withdrawn from the left anterior cerebral artery and the right internal carotid artery to permit reperfusion. Following surgery, the rats were transferred to an intensive care incubator (constant temperature of 37°C) until they awoke completely. Subcutaneous injections of ketoprofen were provided for postoperative care. Certain animals were subjected to sham surgery using the same procedure without arterial occlusion.

### Grouping

Animals were randomly assigned to five groups (n=60 per group): Hypertension (RHRSP), sham surgery (RHRSP + sham surgery), ischemia (RHRSP + MCAO), EA stimulation [EA treatment at the GV20 (Baihui) and GV14 (Dazhui) acupoints for 30 min daily following the induction of MCAO and RHRSP] and sham stimulation (no EA current stimulation after RHRSP + MCAO). Each group was further divided into four subgroups with reperfusion times of one, seven, 14 and 28 days following MCAO (n=15 in each group).

### Sectioning, Nissl staining and immunohistochemistry

Animals were anesthetized with 10% chloral hydrate (0.4 ml/kg) at day one, seven and 14 after MCAO, and transcardially perfused with 200 ml ice-cold phosphate-buffered saline followed by 300 ml formaldehyde (10%). The brains and spinal cords were removed and fixed for 24 h. Following dehydration in graded ethanol and xylene, brain slices were embedded in paraffin, sectioned (Jung Histocut, Model 820-II; Leica, Solms, Germany) to 4 μm in thickness, dewaxed, rehydrated and stained with 1% toluidine blue. Following rinsing, sections were dehydrated in increasing concentrations of ethanol, cleared in xylene and mounted with Permount cover slips.

Normal cells were identified by the presence of Nissl substance in the cytoplasm, loose chromatin and prominent nucleoli. Damaged neurons were identified by the loss of Nissl substance, cavitation around the nucleus and by the presence of pyknotic homogenous nuclei.

Adjacent sections in these groups were set aside for immunohistochemistry with anti-glial fibrillary acidic protein (GFAP) and amyloid precursor protein (APP), as previously described (16). Briefly, sections were incubated with the primary antibody for GFAP (1:500, Santa Cruz Biotech, Santa Cruz, CA, USA) or APP (1:200, Santa Cruz Biotech). After rinsing, the sections were incubated with biotinylated secondary antibodies (1:200, Santa Cruz Biotech) followed by avidin-biotin-peroxidase (Vectastain Elite ABC kit, Vector Laboratories, Inc., Burlingame, CA, USA; 1:200 dilution). Immunoreactivity was visualized with 0.05% diaminobenzidine (DAB) containing 0.03% H_2_O_2_.

### Western blot analysis

Protein samples (50 μg) were loaded on 12% sodium dodecyl sulfate-polyacrylamide gel electrophoresis gels and blotted onto polyvinylidene difluoride membranes. Blots were probed with primary antibodies against Nogo-A (1:1,000; Abnova, Taipei, Taiwan), NgR1 (1:1,000; Millipore Corporation, Billerica, MA, USA) and β-actin (1:2,000; Shanghai Genomics, Shanghai, China) at 4°C overnight, and then incubated at room temperature for 1 h with horseradish peroxidase-conjugated anti-rabbit, anti-mouse and anti-goat secondary antibodies. Signals were detected by chemiluminescence (17). The intensity of each band was calculated with Software ImageJ-1.38× (ImageJ, Bethesda, MD, USA) according to the pixels of the bands in the images.

### Quantitative polymerase chain reaction (qPCR) analysis

Using a standard method with minor modifications, mRNA levels of Nogo-A and NgR1 were measured by qPCR (18). Total RNA was extracted using the Qiagen RNeasy Mini kit (Qiagen Sciences, Inc., Germantown, MD, USA) and was used as template to obtain cDNA by reverse transcription with the Superscript II RNase H-Reverse Transcriptase (Invitrogen Life Technologies, Carlsbad, CA, USA). The following gene-specific primers were used for the qPCR amplifications: Nogo-A forward, 5′-GTCCTGCTTGAAACTGCT-3′ and reverse, 5′-CTTTCGGTTGCTGAGGTA-3′; NgR1 forward, 5′-TGCTGGCATGGGTGTTATGG-3′ and reverse, 5′-CGGAAGGTGTTGTCGGGAAG-3′; β-actin forward, 5′-GGTAAAGACCTCTATGCCAAC-3′ and reverse, 5′-CGGACTCATCGTACTCCTGCT-3′. qPCR was performed with the Prism 7000 Sequence Detection System (Applied Biosystems, Inc., Foster City, CA, USA) and data were analyzed according to the comparative threshold cycle method using glyceraldehyde-3-phosphate dehydrogenase expression for sample normalization. Melting curves for each reaction were generated to ensure the purity of the amplification products.

### Statistical analysis

All data are expressed as the mean ± SD. Multiple group comparisons were conducted by one-way analysis of variance, with a post-hoc Dunnett test for two-group comparisons within the multiple groups. Two-group comparisons were performed using the unpaired Student’s t-test. All statistical analyses were performed using SPSS software, version 13.0 (SPSS, Inc., Chicago, IL, USA), where P<0.05 was considered to indicate a statistically significant difference.

## Results

### EA attenuated neuronal loss in the cervical spinal cord following cerebral ischemia in RHRSP rats

To explore the neuroprotective role of EA in the cervical spinal cord during cerebral ischemia, Nissl immunocytochemistry was performed to determine the neuronal loss in RHRSP rats. As shown in Table I, the number of intact neurons per mm^2^ in the cervical spinal cord of the ischemia group (15.0±1.2) decreased significantly at day 48 following MCAO, when compared with that in the hypertension group (26.1±1.8; P<0.05). EA stimulation reduced this neuronal loss, with a neuron density of 21.3±1.6 (P<0.05, vs. ischemia group). Therefore, stimulating the GV20 (Baihui) and GV14 (Dazhui) acupoints with EA attenuated cervical spinal cord neuronal loss following cerebral ischemia in RHRSP rats.

### EA reduced the expression of GFAP and APP in the cervical spinal cord following cerebral ischemia in RHRSP rats

In order to explore the underlying neuroprotective mechanisms of EA treatment on remote injury in the cervical spinal cord following cerebral ischemia in RHRSP rats, the expression levels of the glial marker, GFAP, and ischemia-induced APP were investigated in the cervical spinal cord. The expression levels of GFAP and APP in the ischemia group increased significantly when compared with those in the sham surgery group (P<0.05) at days 14 and 28 following MCAO, whereas there was no difference between these groups at days 1 and 7. As shown in Fig. 1, the EA treatment reduced GFAP and APP expression levels at day 14 and 28 following MCAO in ischemic rats.

### EA reduced the elevation of Nogo-A and NgR1 expression levels in the cervical spinal cord following cerebral ischemia in RHRSP rats

Protein expression levels of Nogo-A and NgR1 were analyzed in the cervical spinal cord to further investigate the neuroprotective mechanisms of EA. The Nogo-A and NgR1 expression levels in the ischemia group were higher at day 14 and 28 following MCAO compared with those in the hypertension group (P<0.05; Tables II and III), however, these increases in Nogo-A and NgR1 expression were attenuated by the EA treatment (P<0.05, vs. ischemia group).

In addition, qPCR was used to determine the mRNA expression levels of Nogo-A and NgR1 in these models. As shown in Table IV, the mRNA expression levels of Nogo-A in the ischemia group increased at day 28, but not at days one, seven and 14 following MCAO (P<0.05, vs. hypertension group). The NgR1 mRNA expression levels exhibited a similar expression pattern (Table V). EA treatment decreased NgR1 and Nogo-A mRNA expression levels at day 28 (P<0.05, vs. ischemia group). Thus, EA reduced the elevated mRNA and protein expression levels of Nogo-A and NgR1 in the cervical spinal cord following cerebral ischemia in RHRSP rats.

## Discussion

In the present study, it was shown for the first time, to the best of our knowledge, that EA stimulation at GV20 (Baihui) and GV14 (Dazhui) significantly attenuates cerebral ischemia-induced remote cervical spinal cord neuronal loss and changes in GFAP, APP, Nogo-A and NgR1 expression in hypertensive rats. Previously, EA has been shown to significantly ameliorate neurological deficits and cerebral infarction in cerebral I/R-injured rats (19), lessen hippocampal apoptosis in mouse cerebral I/R injury (20) and protect the spinal cord in I/R injured rabbits (21). The results of the present study add to the increasing evidence that EA is an effective therapeutic strategy for various neurological deficits. In addition, the present study has demonstrated a specific role for EA in the treatment of remote cervical spinal cord injury induced by cerebral ischemia.

GV20 (Baihui) and GV14 (Dazhui) acupoints are closely associated with the brain and spinal cord, and so have been commonly used as targets for stroke treatment in ancient China. These acupoints are characterized as protective against hypoxic-ischemic brain damage in immature rats (22) and have been shown to facilitate the recovery of post-ischemic behavioral dysfunction (10). Furthermore, EA pretreatment at these two acupoints has been shown to increase the expression levels of brain-derived neurotrophic factor (BDNF) in the brain tissue and stromal-derived factor-1α in the plasma (23). These observations may provide insight into the neuroprotective mechanism of EA stimulation at GV20 and GV14 in cerebral ischemia.

Astrocytes play an important role in maintaining the neuronal environment and are characterized as being crucial for neuron survival (24). GFAP mainly functions in the regulation of neuron construction and substance metabolism, as well as in the transportation of nervous active amino acids. In addition, GFAP contributes to the recombination events involving the cytoskeleton and the blood-brain barrier, which maintain myelinogenesis and regulate signal transduction. The reactive hyperplasia and hypertrophy of astrocytes can be induced by ischemia and hypoxia, which aids the phagocytosis of harmful ectocytic neuromediators, thus, maintaining the stability of the internal environment and the survival and plasticity of neurons (25). Although the role of GFAP in reactive astrocytes remains unclear, it has been demonstrated that a knock-out of the GFAP gene in mice leads to significantly larger cortical infarct volumes and a more extensive and profound reduction in cortical cerebral blood flow following ischemia (26). Collectively, these observations indicate that astrocytes play an important role in ischemic brain damage. The current study showed that a positive correlation exists between increasing increments in GFAP-positive astrocytes and ischemia-induced APP in the cervical spinal cord following cerebral ischemia; moreover, this increase was significantly attenuated by EA stimulation. Thus, EA appears to not only protect against increases in APP, but also protect against reductions in astrocyte activation, indicating a close association between these two events.

Nogo-A, which is produced by oligodendrocytes, functions as a major myelin growth inhibitory protein and blocks central nervous system (CNS) regeneration (5). Anti-Nogo-A antibody and NgR1 antagonist (NEP1-40) have been shown to improve functional recovery in animals following spinal cord injury or stroke, by neutralizing the inhibitory action of Nogo-A (27,28). However, these results were contradicted by an additional study that demonstrated a marked absence of enhanced Nogo-A expression following CNS injury. Instead, Nogo mRNA expression levels were found to be reduced and Nogo protein expression levels were shown to be moderately upregulated following traumatic lesions in the cortex or in the spinal cord; NgR1 appeared unchanged (29). In the current study, protein expression levels of Nogo-A and NgR1 increased in the cortex within hours of focal cerebral ischemia, and EA suppressed the expression of Nogo-A and NgR1. In addition, following an ischemic event, EA was shown to reduce the expression levels of Nogo-A and NgR1. With this function, EA may contribute to the inhibition of regeneration, immediately after injury prior to glial scar formation.

EA treatment has been reported to reduce the volume of brain infarction and improve the outcome in animal models of focal or global cerebral ischemia (9,10,19). However, the mechanisms of EA-induced brain protection remain unknown, although several theories have been hypothesized in recent years. For example, EA treatment was shown to induce BDNF expression (23), decrease cerebral edema (10), regulate brain metabolites (30) and inhibit apoptosis (9). In the current study, EA was further demonstrated to markedly reduce cervical spinal cord cell loss following cerebral ischemia injury. Simultaneously, EA was also shown to suppress the expression of GFAP and APP and to abolish the enhanced expression of Nogo-A and NgR1. These observations indicate that EA may not only inhibit cell death, but may also enhance neuronal plasticity following cerebral ischemia.

In conclusion, the current study provides novel insights into the neuroprotection afforded by EA treatment on cervical spinal cord injury following cerebral ischemia in hypertensive rats. A possible mechanism may be that EA induces neuroprotection by inhibiting a process that involves astrocyte activation, APP, Nogo-A and NgR1 expression and neuronal loss. These observations indicate a new mechanism of EA, which may also represent a target for a novel therapeutic strategy by which cerebral ischemia-induced remote injury may be attenuated in hypertensive rats.

## Figures and Tables

**Figure 1:** Effects of EA on the expression levels of GFAP and APP in the cervical spinal cord following cerebral ischemia in RHRSP rats; magnification, ×20. Representative immunohistochemical staining images showing (A–F) GFAP-positive and (G–L) APP-positive cell expression at day 14 and 28 after MCAO in the cervical spinal cord of rats that received sham or EA stimulation. EA, electroacupuncture; GFAP, glial fibrillary acidic protein; APP, amyloid precursor protein; RHRSP, stroke-prone renovascular hypertensive; MCAO, middle cerebral artery occlusion.

**Table I:** Number of Nissl stained cells per mm^2^ in the cervical spinal cord at various time points following MCAO (mean ± SD).

Group	Day 1	Day 7	Day 14	Day 28
Hypertension	25.93±1.67	29.27±2.87	26.60±1.21	26.07±1.78
Sham surgery	25.70±1.90	27.37±2.12	28.03±1.11	27.20±1.28
Ischemia	27.35±1.09	29.02±1.06	26.35±1.20	15.02±1.18^a^
EA stimulation	25.82±2.07	29.15±1.85	27.48±1.26	21.32±1.60^b^
Sham stimulation	26.83±1.15	30.17±1.33	26.17±1.35	16.17±1.05

a P<0.05, vs. hypertension group;

b P<0.05, vs. ischemia group; (n=15 per group).

MCAO, middle cerebral artery occlusion; EA, electroacupuncture.

**Table II:** Expression of Nogo-A positive cells in the cervical spinal cord at various time points following MCAO (mean ± SD).

Group	Day 1	Day 7	Day 14	Day 28
Hypertension	1.091±0.318	1.121±0.326	1.113±0.228	1.124±0.268
Sham surgery	1.110±0.204	1.136±0.238	1.117±0.122	1.142±0.286
Ischemia	1.131±0.418	1.156±0.324	1.229±0.375^a^	1.242±0.182^a^
EA stimulation	1.112±0.226	1.144±0.229	1.174±0.273^b^	1.197±0.312^b^
Sham stimulation	1.117±0.217	1.146±0.234	1.210±0.298	1.230±0.405

a P<0.05, vs. hypertension group;

b P<0.05, vs. ischemia group; (n=15 per group).

MCAO, middle cerebral artery occlusion; EA, electroacupuncture.

**Table III:** Expression of NgR1 positive cells in the cervical spinal cord at various time points following MCAO (mean ± SD).

Group	Day 1	Day 7	Day 14	Day 28
Hypertension	1.239±0.270	1.253±0.285	1.246±0.375	1.273±0.263
Sham surgery	1.228±0.388	1.229±0.229	1.235±0.211	1.265±0.294
Ischemia	1.236±0.280	1.226±0.321	1.325±0.239^a^	1.358±0.274^a^
EA stimulation	1.244±0.375	1.234±0.279	1.294±0.293^b^	1.315±0.227^b^
Sham stimulation	1.241±0.295	1.238±0.204	1.311±0.370	1.344±0.311

a P<0.05, vs. hypertension group;

b P<0.05, vs. ischemia group; (n=15 per group).

MCAO, middle cerebral artery occlusion; EA, electroacupuncture.

**Table IV:** Nogo-A mRNA expression levels in the cervical spinal cord at various time points following MCAO (mean ± SD).

Group	Day 1	Day 7	Day 14	Day 28
Hypertension	0.221±0.049	0.254±0.035	0.251±0.041	0.232±0.048
Sham surgery	0.227±0.038	0.250±0.043	0.255±0.036	0.242±0.040
Ischemia	0.276±0.044	0.285±0.032	0.272±0.039	0.451±0.062^a^
EA stimulation	0.238±0.047	0.245±0.033	0.259±0.043	0.319±0.049^b^
Sham stimulation	0.267±0.045	0.265±0.044	0.261±0.038	0.428±0.065

a P<0.05, vs. hypertension group;

b P<0.05, vs. ischemia group; (n=15 per group).

MCAO, middle cerebral artery occlusion; EA, electroacupuncture.

**Table V:** NgR mRNA expression levels in the cervical spinal cord at various time points following MCAO (mean ± SD).

Group	Day 1	Day 7	Day 14	Day 28
Hypertension	0.347±0.052	0.332±0.051	0.353±0.069	0.357±0.063
Sham surgery	0.356±0.058	0.344±0.049	0.342±0.061	0.363±0.054
Ischemia	0.387±0.048	0.383±0.039	0.379±0.065	0.366±0.078^a^
EA stimulation	0.334±0.075	0.336±0.059	0.361±0.035	0.351±0.057^b^
Sham stimulation	0.364±0.055	0.374±0.041	0.368±0.044	0.303±0.081

a P<0.05, vs. hypertension group;

b P<0.05, vs. ischemia group; (n=15 per group).

MCAO, middle cerebral artery occlusion; EA, electroacupuncture.
